The article "Application of Anabaena azotica- and Chlorella pyrenoidosa-Based Algal Biotechnology in Green Production of Algae-Rich Crataegi fructus" was published in 2022. Journal: J Healthc Eng.

# Application of *Anabaena azotica*- and *Chlorella pyrenoidosa*-Based Algal Biotechnology in Green Production of Algae-Rich *Crataegi fructus*

**DOI:** 10.1155/2022/8424890

**Published:** 2022-03-30

**Authors:** Kangjie Wang, Beijuan Hu, Chuangang Zheng, Zhiyi Deng, Jian Duan, Kangxi Qin, Xinwei Cui, Shifeng Li

**Affiliations:** ^1^Yuncheng Agriculture and Rural Bureau of Shanxi Province, Yuncheng 044099, China; ^2^Key Laboratory of Poyang Lake Environment and Resource Utilization, Ministry of Education, Nanchang University, Nanchang 330031, China; ^3^Agriculture Faculty, Xichang University, Xichang 615000, China; ^4^Shanxi Province Jiangxian County Fruit Industry Development Center, Yuncheng 043699, China; ^5^Yuncheng Difulai Biotechnology Development Co Ltd., Yuncheng 043699, China; ^6^Shanxi School-Local Cooperative Microalgae Research Institute, Yuncheng 043699, China; ^7^Vegetation Restoration Engineering Technology Research Center, China Agricultural University, Beijing 100091, China

## Abstract

Nitrogen-fixing *Anabaena* and *Chlorella pyrenoidosa* algal biotechnology are known as new agricultural inputs due to their characteristics and are widely used in the field of agricultural planting. This paper discusses the application of algal biotechnology based on nitrogen-fixing *Anabaena* sp. The advantages of algal biotechnology based on nitrogen-fixing *Anabaena* and *Chlorella pyrenoidosa* in terms of yield, sugar content, polyunsaturated fatty acid content, and high-quality yield of hawthorn were compared.

## 1. Introduction

As for the fruit industry, one of the three major agricultural production industries worldwide [1], its development quality and development level are of great significance to rural revitalization. According to incomplete statistics, the planting area of *Crataegi fructus* has reached 7 million mu in China, accounting for about 10% of the total area of fruit trees planted; the industry scale reached about RMB 20 billion in 2020. *Crataegi fructus*, as a species of edible and medicinal plant, has been widely used in the pharmaceutical industry, food industry and light industry. However, with the continuous expansion of the planting scale, production problems such as the degradation of germplasm resources and increase of group diseases have taken place, especially the significant influence on the quality of *Crataegi fructus* due to the increasing use of fertilizers; therefore, it is urgent to study an ecological, green, efficient, and safe cultivation technology of *Crataegi fructus*, in which, it is quite important to use the new environmentally friendly biotechnology.

Qilipo in Wenxi County and Jiangxian County, Shanxi Province, located in the dominant production area of *Crataegi fructus* in China, have been respectively praised as “The First Village of *Crataegi fructus* Planting in Shanxi” and “The First County of *Crataegi fructus* Planting in China,” both of which have planted about 150,000 mu of *Crataegi fructus* [2]. *Crataegi fructus*, as the local specialty product, is also the product protected by geographical indications of agricultural products and the backbone force for the revitalization of rural industries in the new era. In order to further improve the quality and reduce the use of fertilizers and pesticides, the local government has explored the planting technology of algae-rich *Crataegi fructus* based on *Anabaena azotica* and *Chlorella pyrenoidosa* while relying on the Central Geographical Indication Protection Project, following the “Five-Grade Mode” of the high-quality development of characteristic industries, and focusing on the quality [3]. As confirmed, this mode could significantly increase the yield, the content of unsaturated fatty acid, and sugar content, and also reduce the pesticide residue, thus making the quality of *Crataegi fructus* fundamentally different from that of the fruits in other regions. It is of great significance to create a county-specific brand of *Crataegi fructus* and improve the brand value of the product protected by geographical indications of agricultural products and the industrial competitiveness.

The article "Application of Anabaena azotica- and Chlorella pyrenoidosa-Based Algal Biotechnology in Green Production of Algae-Rich Crataegi fructus" was published in 2022. Journal: J Healthc Eng.

## 2. Selection of Carrier of Biotechnology

Microalgae, a general term for microorganisms, being rich in chlorophyll a and capable of photosynthesis, could absorb heavy metals and inorganic salts from sewage in paddy fields and also degrade organic substances such as pesticides, phenols, and alkanes [4]. The corresponding development and utilization was initiated in the United States, Japan, Germany, Israel, etc. in the 1940s. There are one million species of algae all over the world, over 40,000 of which are known microalgae. At present, the microalgae widely planted or produced with biotechnology mainly include *Chlorella vulgaris*, *Chlorella pyrenoidosa*, nitrogen-fixing blue-green algae, and *Anabaena*. The microalgae could be applied in green production of *Crataegi fructus* based on their own characteristics.

### 2.1. *Anabaena azotica*

#### 2.1.1. Selection Basis

Strong biological nitrogen fixation of *Anabaena azotica* cells: with the nitrogen-fixing method of (N_2_ + 8e^−^ + 16MgATP + 8H^+^⟶2NH_3_ + H_2_ + 16 MgADP +16Pi), azotase contained could fix molecular nitrogen in the air and synthesize amino acids and proteins, thus reducing the plant's demand for nitrogen fertilizers by 10%–30% [5]; it could also dissolve the phosphorus fixed in the soil (Ca_3_(PO_4_)_2_ + CnOnH = H+ + 2PO_4_^3-^ + CnOn - + 3Ca^2+^), and cell secretions can soak into the grid to activate potassium ions for direct absorption by plants so as to prevent the antagonism with other elements in the soil, activate the medium elements and trace elements in the soil, and transport them to the root system, thus promoting the absorption. The rich extracellular polysaccharide colloid EPS and growth stimulating substances could improve soil and improve the fertilizer and water retention capacity of soil.

The article "Application of Anabaena azotica- and Chlorella pyrenoidosa-Based Algal Biotechnology in Green Production of Algae-Rich Crataegi fructus" was published in 2022. Journal: J Healthc Eng.

#### 2.1.2. Mechanism

The reverse carrier system of *Anabaena azotica* cells: The direction of the movement of substances across the membrane is opposite to the direction of ion transfer, namely, when the carrier binds to H+ and then other molecules or ions (such as Na+), they would be transported through the cell membrane in opposite directions. The reverse carrier system could promote the efflux of Na+ and reduce the accumulation of Na+ so as to increase the tolerance of blue-green algae to the salt environment; in addition, it could continuously transfer the extracellular H+ into the cells so as to adjust the balance of the pH value in the cells [6, 7].

### 2.2. *Chlorella pyrenoidosa*

#### 2.2.1. Selection Basis

*Chlorella pyrenoidosa*, the microorganism with the largest surface area in the world, has been praised as the “canned sun” by scientists around the world [8]. It could realize photosynthesis under glimmer poor light, and the effect could be over 10 times the photosynthesis of plants. While being able to greatly improve the accumulation of organic matters in plants, provide rich and balanced natural nutrients, and improve the utilization of water by plants, it could also quickly adsorb various heavy metal ions and promote the excretion of harmful substances from plants. The unique active factor (C.G.F.) could repair the damaged cells, activate phagocytes and interferons, induce plant resistance, degrade the residues of pesticides and fertilizers, and convert them into the useable state beneficial to plants [5, 9].

#### 2.2.2. Mechanism

Photosynthesis mechanism of chlorella (see Figure 1): CO_2_ + H_2_O = (CH_2_O) + O_2_ (conditional enzyme, chlorophyll). At the same time, *Chlorella pyrenoidosa* could make the cellular action of engulf bacteria or viruses active; as the direct user of harmful substances, it could reduce the contents of ammonia nitrogen and nitrite in *Crataegi fructus*. The ability of *Chlorella pyrenoidosa* cells to remove different forms of nitrogen in *Crataegi fructus* can be ordered as follows: ammonia nitrogen > nitrate nitrogen > nitrite nitrogen. The ability to remove different forms of phosphorus can be ordered as follows: orthophosphate > metaphosphate > pyrophosphate > organic phosphate [10].

The article "Application of Anabaena azotica- and Chlorella pyrenoidosa-Based Algal Biotechnology in Green Production of Algae-Rich Crataegi fructus" was published in 2022. Journal: J Healthc Eng.

#### 2.2.3. Kinetic Study

“Severe heavy metal pollution of cultivated land” is one of the practical problems that should be resolved in China at present. The detailed results of the survey on soil pollution of cultivated land indicated that the main pollutants affecting the soil environment and quality of cultivated land were heavy metals, especially cadmium. The study on adsorption kinetics of *Chlorella* indicated that the chemical composition of the cytoderm of *Chlorella pyrenoidosa* had obvious advantages in the adsorption of heavy metals. Cells would continuously release various metabolites into the surrounding environment during growth, such as carbohydrates, amino acids, enzymes, vitamins, organic phosphoric acid, toxins, volatile substances, and inhibitory and promoting factors. As shown in the tracer experiment, at least 5%–10% of the carbon fixed by *Chlorella pyrenoidosa* cells would be released into the waters and soil in the form of DOC, and the value can be up to 10%–25% under better conditions. The adsorption of heavy metals by *Chlorella pyrenoidosa* cells can be ranked as follows: copper > tin > cadmium > nickel > lead > cobalt [11]. By means of active adsorption and passive adsorption, the cells can achieve adsorption and passivation of heavy metal ions, thus solving soil pollution of heavy metals.

## 3. Application Principle of Algae-Rich *Crataegi fructus* Technology Based on *Anabaena azotica* and *Chlorella pyrenoidosa*

### 3.1. Principle of Cell Fission and Oxygenation

The two kinds of cells would be subject to vegetative propagation and geometric fission after entering the soil. One cell would split into billions of cells in the soil, which would continuously release oxygen; the cell fission and reproduction could increase oxygen and ventilate the soil, thus enabling the original beneficial microorganisms multiply and inhibiting the activity of anaerobic bacteria; and bringing soil back to its original state by vital activity of the cells through increasing the organic matters, which can fundamentally solve the problems such as soil compaction, residual and safety, thus ensuring the natural, organic, nontoxic, and harmless nature of agricultural products.

### 3.2. Principle of Nutrient Equalization

The planting pattern of algae-rich *Crataegi fructus* based on *Anabaena azotica* and *Chlorella pyrenoidosa* could provide organic nitrogen, dissolve phosphorus, degrade potassium, and activate the medium and trace elements in the soil, thus promoting rapid growth of *Crataegi fructus* and helping to accumulate nutrients. While effectively promoting photosynthesis and providing comprehensive and balanced nutrients for the growth of *Crataegi fructus*, the organic matters generated could effectively adjust the soil acidity and make it neutral [12]. Active cells, with the phototaxis and chemotaxis, would reproduce by fission after entering the soil, thus promoting soil ventilation and water permeability, providing sufficient oxygen and organic nitrogen for soil, dissolving phosphorus and degrading potassium to activate the medium and trace elements in the soil, and help *Crataegi fructus* to accumulate nutrients. While effectively promoting photosynthesis, they could also provide comprehensive and balanced nutrients for the growth of *Crataegi fructus*, thus improving the quality, reduce the use of fertilizer, and realize high yield.

The article "Application of Anabaena azotica- and Chlorella pyrenoidosa-Based Algal Biotechnology in Green Production of Algae-Rich Crataegi fructus" was published in 2022. Journal: J Healthc Eng.

### 3.3. Principle of Metabolic Promotion

Terpenoids are widely distributed in nature, which could effectively improve the physiological activity of plants in growth metabolism. The planting pattern of algae-rich *Crataegi fructus* based on *Anabaena azotica* and *Chlorella pyrenoidosa* could assist in initiating plant secondary metabolism via the pathway of isoprene pyrophosphate, thus producing terpenoid polymers, which could increase the tolerance of plants to diseases, damage, drought, waterlogging, cold, and continuous cropping, and improve the quality of *Crataegi fructus*. Their application in the planting of *Crataegi fructus* could prolong the shelf life (due to the rich dry matters and increased soluble solids), make the appearance bright, and size uniform.

## 4. Selection of Manufacturers of Biological Fertilizers and Biotechnology

Yuncheng Biotechnology Development Co., Ltd. is a subsidiary of Microalgae Biological Times (Jilin) Ecological Technology Co., Ltd., a high-tech company integrating R&D, production and sales of algal active cell biological fertilizers. It takes the lead in R&D and application of nitrogen-fixing biological products and has three core technologies, namely metrocyte extraction, culture medium, and cell embedding. The development and application technology of algal active cell compound biofertilizers was evaluated as “domestic leading” by the Science and Technology Development Center of the Ministry of Agriculture, and listed as the main promotion technology by the Ministry of Agriculture in 2015. The production of *Anabaena azotica* and *Chlorella pyrenoidosa*-based biofertilizers adopts the single-cell rapid propagation technology. *Anabaena azotica* and *Chlorella pyrenoidosa* were respectively extracted under the microscope and cytoarchitecture analysis was performed, to select the optimal single-cell chain meeting the requirements as the metrocyte chain. After incubating in test tubes for 5–10 days, the cells were inoculated into a 100 ml flask for cultivating for 5–10 days and then inoculated into an 1-liter triangular flask for cultivating for 5–10 days, a 5-liter triangular flask for cultivating for 5–10 days, a 18-liter barrel for cultivating for 10–20 days, and a 1-ton barrel for cultivating for 20–100 days. The whole process was expanded step by step, with continuous illumination and constant temperature; the water and air should be filtered and purified to the required standard; finally, the amount of *Anabaena azotica* and *Chlorella pyrenoidosa* in biological fertilizers reached 8 million/ML, respectively.

The article "Application of Anabaena azotica- and Chlorella pyrenoidosa-Based Algal Biotechnology in Green Production of Algae-Rich Crataegi fructus" was published in 2022. Journal: J Healthc Eng.

## 5. Planting Experiment of Algae-Rich *Crataegi fructus* Based on *Anabaena azotica* and *Chlorella pyrenoidosa* in Wenxi County

### 5.1. Experiment Site and Farmer Information

*Site: Duihou Village, Wenxi County, Shanxi Province* (*experimental field of Wenxi County Half-mountain Crataegi fructus PlantingCooperative*) (see Figures 2–4).

Name and contact information of the farmer: Li Yuxian, 13834397137.

### 5.2. Experimental Design

In the treatment group, the soil was treated with *Anabaena azotica* and *Chlorella pyrenoidosa*, and in the control group, the *Crataegi fructus* plants were managed according to the management procedures of *Crataegi fructus* in Wenxi County. After the experiment, the results were compared by soil analysis and quality analysis. In order to ensure the accuracy of experimental results, during the whole growth process, soil tillage, weeding, irrigation, and pest control were carried out normally.

The *Crataegi fructus* experiment set a treatment group and a control group (covering an area of 1 mu), and the experiment was repeated for 3 times. The soil experiment set a treatment group and a control group (covering an area of 1 mu), and the experiment was also repeated for 3 times.

In each treatment and control group, all fruits of the trees in the east, west, south, north, and middle of the field were collected to determine the sugar content, polyunsaturated fatty acids and high-quality fruit rate; and the soil (1,000 cm^3^) under these trees was collected for analysis.

### 5.3. Experimental Materials

#### 5.3.1. Materials

“Dajinxing” *Crataegi fructus* in Duihou Village, Wenxi County, and the soil collected from the field of *Crataegi fructus* in Duihou Village, Wenxi County.

#### 5.3.2. Experimental Materials

*Anabaena azotica*- and *Chlorella pyrenoidosa*-based biofertilizers were provided by Yuncheng Difulai Biotechnology Co., Ltd., with the single-cell rapid propagation technology, and *Anabaena azotica* and *Chlorella pyrenoidosa* cells reached 8 million/ML, respectively.

The article "Application of Anabaena azotica- and Chlorella pyrenoidosa-Based Algal Biotechnology in Green Production of Algae-Rich Crataegi fructus" was published in 2022. Journal: J Healthc Eng.

### 5.4. Type of Experimental Treatment

### 5.5. Results and Analysis

As shown in Tables 1–3, for *Crataegi fructus* with 200 ml *Anabaena azotica* and *Chlorella pyrenoidosa*, the content of unsaturated fatty acid increased by 0.0041 g/100 g and the sugar content by 1.8% as compared with the control group.

As shown in Table 4, the content of organic matters was increased by 0.18% in soil treated with 400 ml *Anabaena azotica* and *Chlorella pyrenoidosa*.

## 6. Experiment Effect of Algae-Rich *Crataegi fructus* Based on *Anabaena azotica* and *Chlorella pyrenoidosa* in Jiangxian County

### 6.1. Experiment Site and Farmer Information

*Site: Zhengchai Village, Jiangxian County, ShanxiProvince* (see Figures 5–7).

Name and contact information of the farmer: Liu Shanfu 13934396508.

### 6.2. Experimental Materials

#### 6.2.1. Materials

“Dajinxing” *Crataegi fructus* in Zhengchai Village, Jiangxian County, and the soil collected from the field of *Crataegi fructus* in Zhengchai Village, Jiangxian County.

#### 6.2.2. Experimental materials

*Anabaena azotica*- and *Chlorella pyrenoidosa*-based biofertilizers were provided by Yuncheng Difulai Biotechnology Co., Ltd., with the single-cell rapid propagation technology, and *Anabaena azotica* and *Chlorella pyrenoidosa* cells reached 8 million/ML, respectively.

### 6.3. Experimental Design

The *Crataegi fructus* experiment set two treatment groups and a control group (covering an area of 1 mu), and the experiment was repeated for 3 times. The soil experiment set two treatment groups and a control group (covering an area of 1 mu), and the experiment was also repeated for 3 times. In order to ensure the accuracy of experimental results, during the whole growth process, soil tillage, weeding, irrigation, and pest control were carried out normally.

In each treatment and control group, all fruits of the trees in the east, west, south, north, and middle of the field were collected to determine the sugar content, polyunsaturated fatty acids, and high-quality fruit rate; and the soil (1,000 cm^3^) under these trees was collected for analysis.

### 6.4. Type of Experimental Treatment

### 6.5. Results and Analysis

As shown in Tables 5–7, for *Crataegi fructus* with *Anabaena azotica* and *Chlorella pyrenoidosa*, the content of unsaturated fatty acid increased by 0.0054 g/100 g and 0.00845 g/100 g, the contents of diflubenzuron and chlordimeform decreased, and the sugar content increased by 0.45% and 0.80% as compared with the control group.

As shown in Table 8, the contents of organic matters were increased by 0.17% and 0.46% in soil treated with *Anabaena azotica* and *Chlorella pyrenoidosa* as compared with the control group.

The article "Application of Anabaena azotica- and Chlorella pyrenoidosa-Based Algal Biotechnology in Green Production of Algae-Rich Crataegi fructus" was published in 2022. Journal: J Healthc Eng.

## 7. Conclusion

### 7.1. Experimental Results

In conclusion, the one-year experiment on ‘Dajinxing' treated with *Anabaena azotica* and *Chlorella pyrenoidosa* indicated that the use of *Anabaena azotica* and *Chlorella pyrenoidosa* could significantly reduce the pesticide residue on fruits; improve the appearance and quality of the fruits more significantly as compared with those with the use of chemical fertilizers; increase the content of unsaturated fatty acid, and improve the content of nutrients in the fruits; and obviously increase the content of organic matters in the soil.

### 7.2. Benefit Estimation

Within the growth cycle of *Crataegi fructus*, fertilization is generally performed twice (base fertilizer + flushing fertilize), with the average fertilizer cost of 500 yuan/mu/year; pesticides are generally sprayed for about 7 times, with the average cost of 350 yuan/mu/year (50 yuan each time); irrigation is generally performed for 4 times, with the average cost of 160 yuan/mu/year (40 yuan each time); therefore, the total cost is 1,100 yuan/mu/year. The cost of algal active cell biological fertilizer is 120 yuan/mu, and as calculated based on the reduction of fertilizers and pesticides by 30% (850×30% = 255), it can help the farmers to reduce the cost of 255–120 = 135 yuan per mu. The experimental results in 2020 and 2021 indicated that after using *Anabaena azotica* and *Chlorella pyrenoidosa*, the *Crataegi fructus* fruits were relatively uniform in size and good in color, and there were much more high-quality fruits. The average yield of 1,500 kg/mu in the experimental area, and the proportion of high-quality fruits without the use of biological fertilizer was about 85%; based on the unit price of high-quality fruits and non-high-quality fruits in the past two years, the benefit of *Crataegi fructus* per mu was 2,685 yuan. After using *Anabaena azotica* and *Chlorella pyrenoidosa*, the proportion of high-quality fruits increased to 90%, and the benefit was 2,790 yuan per mu. Therefore, the application of *Anabaena azotica* and *Chlorella pyrenoidosa* could reduce the cost of 135 yuan and increase the benefit of 105 yuan, with the total cost saving and efficiency increase of about 240 yuan. As calculated based on the area of 150,000 mu in the project area, the direct economic benefit of 36 million yuan could be increased each year. If calculated based on the area of 7 million mu in 2020, the economic benefit of cost saving and efficiency increase would be about 1.68 billion yuan as conservatively estimated; the specific benefits will be further verified and improved in subsequent promotion experiments.

The article "Application of Anabaena azotica- and Chlorella pyrenoidosa-Based Algal Biotechnology in Green Production of Algae-Rich Crataegi fructus" was published in 2022. Journal: J Healthc Eng.

### 7.3. Recommendations for Future Studies

In future, we will focus on the effects of nitrogen-fixing *Anabaena* and *Chlorella pyrenoidosa* on other fruits such as cherry, apple, and strawberry. If nitrogen-fixing *Anabaena* and *Chlorella pyrenoidosa* do have obvious improvement of content of polyunsaturated fatty acid on other fruits, it will have significant influence on the establishment of Chinese innovative fruit bands.

## Figures and Tables

**Figure 1:** Photosynthesis of *Chlorella*.

**Figure 2:** Wenxi experimental field (overall field and performance of Dajinxing treated with biological fertilizers).

**Figure 3:** Wenxi experimental field (variety performance of Dajinxing treated with biological fertilizers).

**Figure 4:** Wenxi experimental field (variety performance of Dajinxing without being treated with biological fertilizers).

**Figure 5:** Jiangxian experimental field (immature Dajinxing treated with biological fertilizers).

**Figure 6:** Appearance of “Dajinxing” treated with biological fertilizers.

**Figure 7:** Appearance of “Dajinxing” without being treated with biological fertilizers (control group).

**Table 1:** Treatment of *Crataegi fructus*.

Treatment	Experiment treatment comparison
Treatment	*Anabaena azotica* and *Chlorella pyrenoidosa* + 70% conventional fertilization, once on August 1, 200 ml each of *Anabaena azotica* and *Chlorella pyrenoidosa*
Control	Conventional fertilization

**Table 2:** Soil treatment.

treatment	Experiment treatment comparison
Treatment	*Anabaena azotica* and *Chlorella pyrenoidosa* + 70% conventional fertilization, once on August 1, 400 ml each of *Anabaena azotica* and *Chlorella pyrenoidosa*
Control	Conventional fertilization

**Table 3:** *Crataegi fructus* results and analysis.

Item	Unsaturated fatty acid (g/100 g)	Sugar content (%)	High-quality fruit rate (%)
Treatment			
Treatment	0.0583	17.6	90
Control	0.0542	15.8	85

The detection method of unsaturated fatty acid adopted the first method in GB 5009.168–2016 and that of sugar content adopted the method in GB/T 10786–2006; the fruit greater than 0.15 kg was regarded as a high-quality fruit.

**Table 4:** Soil results and analysis.

Item	Sample state	Organic matter (%)
Treatment		
Treatment	Yellowish-brown	1.36
Control	Yellowish-brown	1.18

The detection of organic matters in the soil was performed according to the soil organic matter detection method in NY/T 85–1988 with 50 ml burettes.

**Table 5:** Treatment of *Crataegi fructus*.

Treatment	Experiment treatment comparison
Treatment 1	*Anabaena azotica* and *Chlorella pyrenoidosa* + 70% conventional fertilization, once on July 6, 200 ml each of *Anabaena azotica* and *Chlorella pyrenoidosa*.
Treatment 2	*Anabaena azotica* and *Chlorella pyrenoidosa* + 70% conventional fertilization, once on July 6, 400 ml each of *Anabaena azotica* and *Chlorella pyrenoidosa*.
Control	Conventional fertilization.

The article "Application of Anabaena azotica- and Chlorella pyrenoidosa-Based Algal Biotechnology in Green Production of Algae-Rich Crataegi fructus" was published in 2022. Journal: J Healthc Eng.

**Table 6:** Soil treatment.

Treatment	Experiment treatment comparison
Treatment 1	*Anabaena azotica* and *Chlorella pyrenoidosa* + 70% conventional fertilization, once on July 6, 200 ml each of *Anabaena azotica* and *Chlorella pyrenoidosa*.
Treatment 2	*Anabaena azotica* and *Chlorella pyrenoidosa* + 70% conventional fertilization, once on July 6, 600 ml each of *Anabaena azotica* and *Chlorella pyrenoidosa*.
Control	Conventional fertilization.

**Table 7:** *Crataegi fructus* results and analysis.

Item	Unsaturated fatty acid (g/100 g)	Diflubenzuron (mg/kg)	Chlordimeform (mg/kg)	Sugar content (%)	High-quality fruit rate (%)
Treatment					
Treatment 1	0.04430	Not detected	Not detected	15.25	91
Treatment 2	0.04735	Not detected	Not detected	15.60	90
Control	0.03890	0.0235	0.00981	14.80	84

Not detected indicated that the value was below the detection limit. The detection method of unsaturated fatty acid adopted the first method in GB 5009.168–2016, which of diflubenzuron and chlordimeform adopted the method in GB/T 20769–2008, and that of sugar content adopted the method in GB/T 10786–2006; the fruit greater than 0.15 kg was regarded as a high-quality fruit.

**Table 8:** Soil results and analysis.

Item	Sample state	Organic matter (%)
Treatment		
Treatment 1	Yellowish-brown	1.43
Treatment 2	Yellowish-brown	1.72
Control	Yellowish-brown	1.26

The detection of organic matters in the soil was performed according to the soil organic matter detection method in NY/T 85–1988 with 50 ml burettes.

## Data Availability

The datasets used and/or analyzed during the current study are available from the corresponding author on reasonable request.
